# Free Radical Production in Immune Cell Systems Induced by Ti, Ti6Al4V and SS Assessed by Chemiluminescence Probe Pholasin Assay

**DOI:** 10.1155/2012/380845

**Published:** 2012-06-19

**Authors:** Sandra C. P. Cachinho, Fanrong Pu

**Affiliations:** Clinical Engineering, University of Liverpool, Liverpool L69 3GA, UK

## Abstract

The oxidative burst of human blood cells in the presence of different metal materials was investigated using chemiluminescence assay. Commercial pure titanium (Ti), titanium alloy (Ti6Al4V), and stainless steel 316L (SS) in particulate form with <20 *μ*m in size were used. The effect of particulate materials opsonisation on the upregulation of the respiratory burst production by blood cells was also assessed. The largest chemiluminescence response was achieved after simultaneous injection of the stimulants fMLP+PMA. Moreover, Ti and SS induced a greater inflammatory reaction compared to Ti6Al4V, since the respiratory burst mounted was higher for both materials after opsonisation treatment. These results suggest that *in vitro* chemiluminescence response and respiratory burst measurements proved to be composition and treatment dependent.

## 1. Introduction

Implanted biomaterials, introduced into the human body, interact initially with blood inducing a nonspecific host defence responses which are critical to their integration and susceptibility to infection [1–4]. Generally, when infection occurs, it tends to be persistent and intractable with antibiotics and the removal of the implant to clear the infection is often required [2, 5].

The body's response to a foreign body is characterised by an initial infiltration of polymorphonuclear leukocytes (PMNs), where neutrophils and monocytes are the first inflammatory cells to be recruited to an implanted surface exposed to blood. These blood cells can subsequently release cytokines and inflammatory mediators, which recruit additional cells—macrophages, fibroblasts, lymphocytes, and endothelial cells—that proliferate and mediate a chronic response [4, 6–8]. Adhesion, chemotaxis, aggregation, and activation in response to the inflammatory stimuli are processes in which cells may go through upon material contact [4, 9]. After adhesion to biomaterial surfaces, different leukocyte reactions such as phagocytosis, respiratory burst (generation of reactive oxygen species, ROS), and protease release may also occur, resulting in the deterioration of the implanted material and injury to peripheral tissue [10, 11]. The production of highly reactive oxygen intermediates (“oxygen burst” or “respiratory burst”) by PMNs, such as superoxide anion (O_2_^−^), hydrogen peroxide (H_2_O_2_), and hydroxyl radical (OH^•^), may be a major source of damage to inflamed tissues and implanted materials degradation [12–14]. These oxidative metabolites are potent bactericides and constitute an important part of the oxygen-dependent bactericidal killing mechanism of the PMNs [12, 15, 16]. The oxidative response is mounted mainly against bacteria to destroy them, but the oxygen radicals are secreted during inflammatory reactions, too; moreover, they have been recently suggested to be mediators of cytokine activity on target cells, mainly for tumour necrosis factor (TNF) and interleukin-8 (IL-8) [16, 17]. 

The adhesion of neutrophils and other leukocytes to implanted surfaces and their activation, with the subsequent release of potential biomaterial and tissue-damaging agents, are important phenomenon in the host response to biomaterials, and whether implanted biomaterials increase the risk for infection is an important issue to be addressed. The NADPH oxidase-mediated respiratory burst is a result of neutrophil activation, which is triggered following occupation of specific receptors on neutrophil surfaces, binding to certain soluble inflammatory molecules or to invading microorganisms. *In vitro* the burst may also be initiated by soluble phorbol myristate acetate (PMA) or N-formyl-methionyl-leucyl-phenylalanine (fMLP) [15, 18, 19]. 

In this work, the effect of three commercial particulate metal materials on leukocyte adhesion and their oxidative response was investigated. Whole blood was used to investigate leukocytes oxidative burst activity in contact to the particulate materials. The aim of this part of the research was to evaluate the potential of particulate materials with different compositions, to directly stimulate nonspecific activation of human inflammatory cells. The respiratory burst activity of cells from whole human fresh blood in the presence of materials was studied using *in vitro* chemiluminescence assay where fMLP and PMA were used as reference activators. Stimulated cell function* in vitro* has been largely studied using isolated peripheral blood mononuclear cells (PBMC); however, in this work, whole blood assay was preferred because of the better approximation to the *in vivo* situation. 

## 2. Materials and Methods

### 2.1. Materials

Spherical pure titanium (Ti), titanium alloy (Ti6Al4V), and stainless steel 316L (SS) in particulate form with <20 *μ*m in size were purchased from Alfa Aesar (UK). Prior to use in cell culture, material particles were sterilised in 70% ethanol followed by washing in PBS and media. For cell culture particles were weighed, from this the number of particles was calculated; a ratio of 1 : 1 particle per cell was used. 

### 2.2. Whole Blood Sample Preparation

Fresh blood was collected from healthy adult volunteers by venous puncture and gently mixed with heparin (20 mL human whole blood gently mixed with 40 *μ*L heparin); informed consent was obtained from each individual enrolled in this study. For chemiluminescence experiments, *20 *μ**L of whole blood was used in each well. 

### 2.3. Chemiluminescence Assay

For the determination of the respiratory burst resulting from cells and biomaterials interaction, pholasin-dependent chemiluminescence was used. Free radicals and other reactive oxygen species produced by activated cells interact with Pholasin, and the luminescent response can be measured. Pholasin is a photoprotein that emits light after excitation with reactive oxygen species.

*20 *μ**L of whole blood was diluted in 2 mL of blood dilution buffer. Duplicate wells were prepared for each material with *90 *μ**L of reconstitution and assay buffer, *20 *μ**L adjuvant-K and *50 *μ**L of Pholasin (all reagents from Abel Cell Activation Test Kits with Pholasin, Knight Scientific Limited, UK) and *20 *μ**L of blood suspension. Two wells without materials were prepared to verify the activation effect of the materials on the cells. Opsonised particles were also used to determine the effect of complement on cells activation. The plate was then placed in the microplate reader FLUOstar OPTIMA (BMG Labtech, UK) previously set to 37°C and automatically shaken for 3 sec at 300 rpm before measurements were started. The microplate reader was controlled by the computer using the OPTIMA program. The program was set such that the luminometer measured light emission from each well every 20 sec. The light output from each well was measured for 40 min. At that time point, *20 *μ**L of each stimulant, formyl-methionyl-leucyl-phenylalanine (fMLP, *12 *μ**mol/L) and phorbol-myristate-acetate (PMA, *8 *μ**mol/L), were injected into each well and the light emitted measured for another 40 min. Luminescence values were plotted as the amount of light emitted versus time. Data were analysed using OPTIMA MARS-data analysis software. 

### 2.4. Graphical Representation and Statistical Analysis

Experiments were repeated for four volunteers, and the means and standard deviations were calculated; this will be expressed as mean ± 1 standard deviation. Statistical significances were evaluated by one-way analysis of variance (ANOVA) and by post hoc Tukey test using Statistical Comparisons Sciences (SPSS) version 16.0 for Windows software. Differences were considered to be statistically significant at *P* < 0.05. All the results are represented in graphical form using Microsoft Excel.

## 3. Results

### 3.1. Chemiluminescence

The results for the oxidative burst analysis of whole blood cells by continuous measurement of the cells chemiluminescence response to Ti, Ti6Al4V and SS particles are shown in Figures 1, 2, and 3, respectively. Each figure shows representative curves of the chemiluminescence response of the cellular interaction with the surface of the particle for a period of 80 min. In the measurement of the oxidative burst activity of blood cells, PMA and fMLP activators were used in combination to maximally stimulate cells. The stimulants were added to the reaction mixture after the blood cells were allowed to interact with the surfaces for 40 min. 

A general trend can be observed in all figures where maximum ROS production was reached between 2700 sec and 3100 sec and after (fMLP+PMA) stimulation. The chemiluminescence response elicited a slight decrease after stimulation and remained constant during the rest of the assay. Low chemiluminescence response was elicited by the particulate materials in the absence of stimulants.

The largest chemiluminescence response was determined for SS, with or without opsonisation (2008 ± 206 and 6077 ± 3008 at 3060 sec for SS and SSops, resp.) (Figure 3), while on the other particulate metals, the response was smaller (1283 ± 379, 3397 ± 901, 485 ± 140, and 1395 ± 372 at 3060 sec for Ti, Tiops, Ti6Al4V, and Ti6Al4Vops, resp.) (Figures 1 and 2). The chemiluminescence response, after (fMLP+PMA) stimulation, was more sustained when blood cells were in contact with Tiops and SSops particulates, indicative of a more prolonged production of oxygen radicals by cells on these materials.

In order to compare ROS production between materials, two specific time points were chosen: one before stimulant injection and the other after stimulant injection at 1800 and 3200 sec, respectively. The results are shown in Figures 4 and 5.  Figure 4 shows the chemiluminescence response of whole blood cells on particulate surfaces prior to the addition of stimulants, while Figure 5 shows the chemiluminescence response subsequent to fMLP+PMA addition. 

With the exception of opsonised SS (5967 ± 2689), after stimulant injection, the highest production of ROS was detected for whole blood cells (negative control) without particulate materials contact (3705 ± 161) when compared with cells in contact with metal particles (≤3402) (Figure 5). Statistical differences (*P* < 0.05) were observed between the negative control and whole blood cells cultured in the presence of particulate Ti and particulate Ti6Al4V. Particulate materials downregulated the chemiluminescence response and a decrease in the respiratory burst activity was demonstrated. 

The lowest ROS production can be observed for all situations before stimulant injection (268 ≤ ROS ≤ 940) (Figure 4) when compared to the response after cell stimulation (468 ≤ ROS ≤ 5967) (Figure 5).

At 1800 sec, similar chemiluminescence levels were detected between Ti and Tiops (853 ± 311 and 847 ± 452, resp.) and Ti6Al4V and Ti6Al4Vops (239 ± 39 and 268 ± 16, resp.), while opsonised SS showed a lower chemiluminescence signal compared to the nonopsonised SS (514 ± 47 and 898 ± 217, resp.) indicating a decrease in the respiratory burst activity (Figure 4). No statistical differences were demonstrated between opsonised and nonopsonised particulate materials, indicative that opsonisation did not affect the production of ROS; however, significant differences (*P* < 0.05) were noted between Ti and Ti6Al4V, Ti6Al4V and SS, and Tiops and Ti6Al4Vops, demonstrating that the respiratory burst activity was material dependent. The respiratory burst activity induced by the presence of particulate Ti6Al4V, opsonised (268 ± 16) and nonopsonised (239 ± 39), was statistically significant when compared to the negative control (whole blood cells: 940 ± 296) and the positive control (whole blood cells+zymops: 819 ± 41), showing lower ROS production. Ti6Al4V particles downregulated the respiratory burst, and no further increase in ROS production was induced by the presence of opsonised particles. No statistical differences were recorded for the other particulate materials composition compared to the negative and positive controls. 

3200 sec after stimulation with PMA+fMLP, the respiratory burst activity was upregulated for all experimental conditions with maximum ROS production observed when whole blood cells were in contact with opsonised SS (5967 ± 2689) (Figure 5). An increase in the ROS production was induced when whole blood cells were in contact with opsonised particulates compared to the amount produced when cells were in contact with nonopsonised ones (from 1290 ± 347, 468 ± 105, and 2000 ± 158 to 3402 ± 746, 1459 ± 454, and 5967 ± 2689 for Ti, Tiops, Ti6Al4V, Ti6Al4Vops, SS, and SSops, resp.), indicating that opsonisation increased the production of oxygen radicals by whole blood cells. Statistical differences, *P* < 0.05, were recorded between Ti and Tiops and between SS and SSops, showing the effect of opsonisation on stimulation of a respiratory burst. No statistical differences were observed between nonopsonised particulate metals. The highest production of ROS observed for opsonised SS was statistically different compared to the other particulate materials, either opsonised or nonopsonised; providing further evidence of material composition effect (Figure 5). Significant differences (*P* < 0.05) were also recorded between opsonised SS and the positive control, whole blood cells cultured with opsonised zymosan, (2481 ± 336) supporting the evidence mentioned above. No differences were observed between the positive control and the other opsonised particulate materials. 

## 4. Discussion

The measurement of chemiluminescence serves as an excellent parameter for the quantitative evaluation of nonspecific leukocytes activation, and it has been widely used as a sensitive and accurate method for the assessment of ROS production [20, 21]. In this study, a chemiluminescence assay was used to evaluate the potential of immune cells to become activated after direct contact with particulate materials of different compositions, opsonised and nonopsonised. The light resulting from the interaction of free radicals, produced by activated cells, with the photoprotein Pholasin was detected and plotted as a function of time. The oxidative burst depends on the activity of NADPH oxidase, a transmembrane electron transport chain that reduces oxygen to superoxide. When PMNs are stimulated by soluble stimulants or phagocytose materials, the multicomponent system of NADPH oxidase is rapidly assembled and activated. [22–24]. There are differences in the final species of released ROS that depends on the type of stimulant and the pathway of activation. The positive references stimulants used in this work to activate the respiratory burst were the receptor stimulant fMLP and the phorbol ester PMA which act through different pathways. fMLP, a formylated oligopeptide, is structurally similar to bacteria-derived peptides. It is a ligand that binds to specific fMLP receptors on the cell surface and acts by means of a mechanism that is dependent on both intra- and extracellular calcium and on a process that includes phospholipase and protease activation. PMA is a chemical that lacks specific cell surface receptors, and so it bypasses this step and activates the specific enzymes involved in the signal transduction sequences (i.e., protein kinase C).

 In this study, the injection of Pholasin into each well did not show any effect on the light detected, showing that whole blood cell-particulate material interaction did not cause any effect on the respiratory burst; this situation, which happened before PMA+fMLP injection, might indicate that materials downregulate the production of ROS or that cells might have been activated at some earlier point in the assay. The production of ROS was also low in unstimulated whole blood cells without particulate materials contact. Unstimulated whole blood cells were expected to generate no measurable or very low amounts of ROS since the NADPH oxidase system should have been inactive at that stage. After simultaneous injection of the stimulants, fMLP+PMA, a peak for the light emitted was observed due to an increase in the production of ROS. This was found in stimulated whole blood cells with and without particulate materials contact. The response after the injection of stimulants was higher in all situations. This was indicative that whole blood cells were not activated by any of the materials tested in this work prior to the addition of PMA+fMLP, since a lower luminescent signal was demonstrated due to the lower production of ROS. *In vitro* evidence [25–27] indicated that macrophages and neutrophils on biomaterial surfaces have a low chemiluminescence response and, in addition, a low capacity to mount an oxidative response when stimulated by a soluble stimulus. It has been also shown that the human PMN function and the respiratory burst *in vitro* are influenced by cell adhesion to a surface. Increased adherence and spreading of PMNs to materials too large to phagocytose can lead to increased activation of oxygen metabolism [1, 28]. Moreover, the protein adsorption to a surface influences the *in vitro* cell attachment and function [25]. Opsonised metal particles induced higher levels of light emitted when compared to the nonopsonised ones. The greatest difference was found for whole blood cells in contact with opsonised stainless steel where the highest light emitted was recorded immediately after fMLP+PMA injection. Furthermore, the data indicated that Ti and SS could induce a greater inflammatory reaction compared to Ti6Al4V, since the respiratory burst mounted was higher for both after opsonisation treatment. If large amounts of H_2_O_2_ and O_2_^−^ are produced *in vivo* when a biomaterial is inserted into the human body, host tissues may be damaged. Titanium has been suggested as a nonreactive material used *in vivo *due to its passive oxide layer; however, the results from this study indicated that cells in contact with opsonised particulate titanium may be stimulated when challenged with fMLP+PMA. The same result was found by Eriksson et al. [9] where PMNs on titanium did not produce ROS spontaneously but were able to elicit a response when exposed to opsonised zymosan. Cells adherent to titanium were not active but have the ability to respond to a microorganism when challenged with the correct stimuli. In another work by Nygren et al. [29], titanium and stainless steel sheets implanted *in vivo* were analysed by chemiluminescence and the ability of the surface-adhering leukocytes to mount a respiratory burst after stimulation with PMA or zymosan was measured. The results from their study showed higher ROS production for stainless steel when challenged with opsonised zymosan when compared with titanium or PMA challenge. This suggests that titanium might not be as inert as previously described and when implanted *in vivo* might complex with serum proteins and induce the production of ROS. 

From this study, the production of ROS was found to be lower when whole blood cells were in contact with nonopsonised particulate metals compared to the opsonised ones. Comparison of the degree of inhibition of stimulated chemiluminescence, resulting from exposure of whole blood cells to various particulate metals, can be summarised as follows: (Ti6Al4V < Ti < SS) < (Ti6Al4Vops < Tiops < SSops), indicating that opsonisation upregulates the production of ROS by immune cells when in contact with those particulate materials; the same effect can be observed even after PMA+fMLP stimulation, resulting in higher respiratory burst activity. 

Some research [28, 30, 31] has shown *in vitro* that PMNs adhering to protein-coated substrates do not produce ROS unless exposed to a stimulus, which is in accordance with the results from this study. Opsonisation did not affect the activation state of cells until PMA+fMLP was injected and the respiratory burst was induced. It has been also published [32–34] that particles coated with serum constituents might make those surfaces less reactive. Serum proteins, for example, albumin, fibrinogen, and hemoglobulin, bind to and change the nature of particulate powder surfaces such that they lose the potential to stimulate cells. It has been suggested [28] that serum provides a mixed protein coating for biomaterials possibly creating a biocompatible interface between materials and cells. Terkeltaub et al. [35] found that the presence of serum in hydroxyapatite (HA) particles incubated with cells or the pretreatment of HA crystals with serum resulted in a marked suppression of neutrophil activation to HA crystals and the superoxide release was reduced. The same results were found by Remes and Williams [33] where serum proteins bound to CaHPO_4_ powders reduced the stimulation of neutrophils. This inhibitory effect was observed in this study where opsonised particles, metals and zymosan, did not affect the respiratory burst activity and the production of ROS was not affected, until challenged with fMLP+PMA. This low peak luminescence was a feature of all opsonised zymosan samples used in this study and was reproducible across different donors. Clearly, long-exposure times before stimulant addition did not affect the response. Besides evidence [24, 36] that zymosan, a yeast particle which is opsonised and commonly used stimulus for chemiluminescence studies, is particularly useful for stimulating neutrophils phagocytosis which results in a chemiluminescent response that can be 10–20 times higher than unstimulated values, some *in vitro* studies showed a reduced capacity of human cells to mount an oxidative response when the cells were challenged with opsonised zymosan [37]. Ginis and Tauber [30] found that nonopsonised zymosan did not stimulate O_2_^−^ generation by neutrophils, but rigorous O_2_^−^ response could be induced in cells adherent to fibronectin. The type of protein bound to a surface might explain the ability for surfaces to stimulate differing respiratory burst effects from cells in direct contact. Surface contact alters neutrophils behavior, and the oxidative burst can be reduced compared to control cells. 

Since macrophages and neutrophils are the major cells presented in blood, that contribute to the respiratory burst, the lower ROS production in the presence of opsonised zymosan, before stimulants addition, might be explained on the experimental evidence mentioned above. Macrophages are far less potent than neutrophils and eosinophils at producing ROS, and they might need time to acquire an activated phenotype to upregulate their bactericidal capability [38].

## 5. Conclusions

The chemiluminescence assay was demonstrated to be a useful technique to understand the interaction of immune cells and implanted materials in terms of reactive oxygen species production, known to be harmful to the tissues and potentially damaging to implanted medical devices. In this study, the stimulatory effects on whole blood cells caused by a series of particulate metals were assessed using the chemiluminescence method based on the photoprotein Pholasin. The results indicated that the exposure of whole blood cells to particulate metal materials could generate a respiratory burst when challenged with fMLP+PMA. ROS production was upregulated in the presence of opsonised particulate metals, where the highest production was found for opsonised stainless steel followed by opsonised titanium; suggesting these materials have the potential to stimulate an inflammatory response directly and consequently activation is directed by protein modification or by complement activation. 

## Figures and Tables

**Figure 1:** Chemiluminescence response of whole blood cells to Ti, opsonised and nonopsonised, and opsonised zymosan (positive control). Reaction mixture included whole blood cells without particulate materials (negative control) and in the presence of Ti, Tiops, and Zymops particles. Cells were stimulated with fMLP+PMA at 2400 s.

**Figure 2:** Chemiluminescence response of whole blood cells to Ti6Al4V, opsonised and nonopsonised, and opsonised zymosan (positive control). Reaction mixture included whole blood cells without particulate materials (negative control) and in the presence of Ti6Al4V, Ti6Al4Vops, and Zymops particles. Cells were stimulated with fMLP+PMA at 2400 s.

**Figure 3:** Chemiluminescence response of whole blood cells to SS, opsonised and nonopsonised, and opsonised zymosan (positive control). Reaction mixture included whole blood cells without particulate materials (negative control) and in the presence of SS, SSops, and Zymops particles. Cells were stimulated with fMLP+PMA at 2400 s.

**Figure 4:** ROS production during whole blood cell interactions to opsonised and nonopsonised particulate materials before fMLP+PMA injection and at 1800 sec of chemiluminescence measurement (reaction mixture included whole blood cells without particulate materials, whole blood cells in the presence of Ti, Ti6Al4V, SS, Tiops, Ti6Al4Vops, SSops, and Zymops particles) (∗, +, ♦ *P* < 0.05).

**Figure 5:** ROS production during whole blood cell interactions to opsonised and nonopsonised particles materials after fMLP+PMA injection and at 3200 sec of chemiluminescence measurement (reaction mixture included whole blood cells without particulate materials, whole blood cells in the presence of Ti, Ti6Al4V, SS, Tiops, Ti6Al4Vops, SSops, and Zymops particles) (∗, +, ♦ *P* < 0.05).

## List of Abbreviations

Ti: Pure titanium
Ti6Al4V: Titanium alloy
SS: Stainless Steel 316L
fMLP: N-Formyl-methionyl-leucyl-phenylalanine
PMA: Phorbol myristate acetate
PMNs: Polymorphonuclear leukocytes
ROS: Reactive oxygen species
PBMC: Peripheral blood mononuclear cells
Ops: Opsonisation.
